# Ladder-Like Low Iodine Delivery Rate Injection Protocols Based on BMI at 70 KV by Automated Tube Voltage Selection in Coronary CTA

**DOI:** 10.1155/2022/7804015

**Published:** 2022-07-16

**Authors:** Shang Ge, Jian-Yao Zhu, Han Liu, Yuan Chen, Zhao-Huan Zhu

**Affiliations:** Department of Radiology, Affiliated Huai'an No 1 People's Hospital of Nanjing Medical University, Nanjing, China

## Abstract

**Objective:**

To evaluate the feasibility of reducing the injection velocity and volume of contrast agent according to BMI, and the effect of body weight (BW), body surface area（BSA）, body mass index（BMI），and blood volume (BV) on aortic contrast enhancement when the voltage of third-generation dual-source CT is selected at 70 KV.

**Methods:**

A total of 280 patients selected at 70 KV were randomly divided into an experimental group and a control group. Each group was divided into 7 subgroups according to BMI ≤20, 20–21, 21-22, 22-23, 23-24, 24-25, and 25–26. The experimental group uses 2.3/2.4/2.5/2.6/2.7/2.8/2.9 ml/s injection speed with 350 mgI/ml contrast agents according to the subgroups; injection time was fixed at 10 s. In the control group, the fixed injection flow rate was 3.5 ml/s, time was 12 s with a total of 42 ml. Subjects in both groups were inspected to adaptive prospective ECG-gating sequence scanning, and subjective and objective image quality of the two groups were compared using Student's *t*-test. BMI, BSA, and BV were calculated from the patient's body weight and height. We assess the relationship between aortic attenuation and BW, BMI, BV, and BSA using regression analysis or correlation analysis.

**Results:**

Significant differences exist in vascular enhancement between the two groups; SNR and CNR of objective image quality in the experimental group were lower than those in the control group (*P* < 0.05). Both groups had the same subjective image scores (*P* > 0.05). The number of vessels in the optimal enhancement range counts more in the experimental group than in the control group (*χ*2 value = 334.25, *P* ＜ 0.05). In the control group, a weak to medium correlation was seen between vascular enhancement and BMI (*r* = −0.20), BW (*r* = −0.42), BSA (*r* = −0.46), and BV (*r* = −0.48) (*P* ＜ 0.05 for all).

**Conclusions:**

Compared to BW, BSA, and BV, a weaker negative correlation exists between vascular enhancement and BMI when ATVS selects 70 KV. However, as a much easier way to operate, the stepped low flow and low-contrast agent injection based on BMI was feasible, and the image quality was more homogenized than that of the control group.

## 1. Introduction

Coronary CT angiography could evaluate the degree of vessel stenosis and plaque. During this process, contrast enhancement is a key element of the quality of the image. The phantom study had proven that low attenuation (<200HU) may result in the overestimation of stenosis while high attenuation (>500HU) leads to underestimation [1]. Therefore, the appropriate degree of vascular enhancement is very important for image diagnosis. Compared with the second-generation dual-source CT, the third-generation dual-source CT's unique dose-care technology, the CARE Dose 4D, will automatically adjust the tube current according to the scan results based on the anatomical level of patients. Meanwhile, CARE KV technology could select tube voltage automatically within 70–120 kV. Quite a number of studies had proved that there is no statistical difference in image quality between low and high tube voltage [2, 3]. However, Wang et al. [4]showed that automatic tube voltage and automatic tube current could not maintain the consistency of image enhancement, and body weight and BMI still had an impact on image quality. In the actual clinical operation, some patients showed excessive vascular enhancement when there is a contrast agent with a fixed volume and flow rate at 70/80 KV. Based on the above situation, this study, on the premise of excluding the influence of tube voltage on contrast agent enhancement, aims to explore the feasibility of a personalized contrast agent scheme under 70 KV based on BMI and the effect of individual factors on the vascular enhancement with fixed the contrast volume.

## 2. Materials and Methods

### 2.1. Patients

From September to December 2021, a total of 280 patients came to the Affiliated Huai'an No.1 People's Hospital of Nanjing Medical University for CCTA. Patients were divided into the experimental and control groups according to the principle of randomness. The data of age, height, weight, and heart rate were collected. There are 140 patients in two groups after screening. Exclusion criteria are as follows: (1) coronary artery bypass grafting or stenting, (2) decompensated cardiac, renal, or hepatic insufficiency, (3) heart valve replacement, and (4) arrhythmias. A total of 158 men and 122 women were enrolled in the study. The study was approved by the institutional review board, and informed consent was obtained from all patients. Patients take beta-blockers to reduce heart rate half an hour before scanning. Then, ECG was connected, and breathing training was performed. Sublingual nitroglycerin 0.5 mg would be administered later. Iohexol (350 mgI/mL) injection was injected intravenously through the right elbow with a high-pressure double-head syringe.

### 2.2. Scan Protocol

All examinations were performed using a third-generation Dual-Source CT Scanner (SOMATOM definition Force; Siemens Healthcare， Forchheim， Germany). DSCT uses an adaptive prospective-gating sequence with tube voltage from 70 to 120kVp. The information of patients was recorded at 70 KV. Bolus tracking was used to trigger data acquisition, and the trigger threshold is set to 60HU above baseline. Gantry rotation speed was 0.25 seconds per rotation and collimation of 96 × 0.5 mm. Axial images were reconstructed at best diastolic and best systolic phases using advanced modeled iterative reconstruction (ADMIRE, Siemens Healthcare, Forchheim, Germany) at strength 3 and a medium soft convolution kernel (Bv36). The scanning window ranges from 1 cm below tracheal bifurcation to the level of the heart diaphragm.

### 2.3. Contrast Agent Injection Program

BMI was calculated according to the collected data on height and weight. After the automatic tube voltage selection at 70kv, patients were divided into 7 subgroups based on the range of BMI (19–26). The 7 subgroups were injected with different rates (2.3∼2.9 ml/s) and volumes (23∼29 ml), and the injection time of the experimental group was fixed at 10s. Then, the saline was injected with the volume of 18 ml, the rate was 3 ml/s, and the time was 6 s. In the control group, the dosage was fixed at 42 mL, 3.5 mL/s, and 12 s. Normal saline was injected at 40 ml, 4 ml/s, and 10s as usual.

### 2.4. Objective Image Quality

The CT value of the aortic root was measured. The ROI area is tried to be as consistent as possible with a diameter of 2 cm. Its SD value was used as the noise level. Coronary vessels were divided into 18 segments based on The Society of Cardiovascular Computed Tomography 2014 [5]. The CT values of the proximal, mid, and distal segments of the right coronary artery (RCA) and left anterior descending artery (LAD) and proximal and distal segments of the left circumflex artery (LCX) were recorded, avoiding the vessel wall and calcified plaques. The right parasternal muscles were used as the signal contrast tissue. The signal-to-noise ratio (SNR) and CNR were calculated according to the following formula: SNR=CT_aortic root_/SD_noise_; CNR=(CT _aortic root_ -CT _contrast tissue_)/SD_noise_. The right parasternal soft tissue was regarded as a contrast tissue. 300–450HU was defined as the optimal artery enhancement range. Experimental and control groups were compared as a whole or as subgroups. Other factors such as body weight（BW）, blood volume（BV）, and body surface area (BSA) were also included in the analysis to figure out the relationship between these factors and vascular enhancement.

The body surface area formula is Mosteller formula:

 
*BSA* *=* *(height(cm)∗weight(kg)/60)^(1/2)* [6]
  Blood volume formula:
  Male BV = 0.3669*∗*height(m)^3 + 0.03219*∗*weight(kg)+0.6041
  Female BV = 0.3561*∗*height(m) ^3 + 0.03308*∗* weight(kg) +0.1833 [7]

### 2.5. Subjective Image Quality

Use a 4-point Likert scale to access the subjective image quality: 4, excellent image quality, defined as a complete absence of motion artifacts; 3, acceptable image quality, not compromising diagnostic vessel assessment; 2, reduced image quality due to motion, noise, or low contrast, but still sufficient to access significant stenosis; 1, nondiagnostic image quality [4]. Two experienced radiologists evaluate the image and a consensus was reached by discussion in case of disagreements.

### 2.6. Statistical Analysis

Statistical analysis was performed using commercially available statistical software (SPSS 25.0; SPSS, Inc., Chicago, IL, USA). A one-way ANOVA was used to detect whether differences exist between BMI subgroups. Further specific differences were performed using the LSD method. Age, height, weight, BMI, heart rate, CNR, SNR, and the injection parameters of the two groups were compared using an independent samples *t*-test or Mann–Whitney *U* test based on conditions. Nonparametric data were evaluated with the Mann–Whitney *U* test. Single or multiple linear regression models were used to investigate the influence of BW, BSA, and BV on enhancement. Statistical significance was accepted at *P* < 0.05.

## 3. Result

### 3.1. Patients Characteristics

There were no significant differences between the experimental and control groups with regard to sex, age, height, weight, heart rate, or BMI. Patient characteristics are summarized in Table 1.

*Correlation between BMI and Vascular Enhancement*. Referring to previous studies [6], the aortic root was taken to judge the difference in vascular enhancement between subgroups with fixed injection volume. The CT values of the aortic root were normally distributed after the KS test (*P* = 0.2 > 0.05). Homogeneity of variance was checked by one-way ANOVA, and Levene's test value = 1.817, *P* = 0.100 > 0.05, so homogeneity of variances was achieved. ANOVA turns out that *F* = 2.372, *P* = 0.03＜0.05， meaning that a difference exists between subgroups based on BMI. Further LSD methods turned out that BMI≤20 subgroup and 20∼21/21∼22/22∼23/23∼24/25∼26 subgroup have a statistical difference, *P*＜0.05 (*P* value = 0.008/0.016/0.049/0.016/0.001. *P* values of other subgroups in pairs were all more than 0.05. Rank correlation analysis was carried out between aortic root vascular enhancement and BMI subgroups in the control group, *P* = 0.016 < 0.05, correlation coefficient *R* = −0.20. ANOVA between the experimental group showed *F* = 0.880, *P* = 0.512 > 0.05.

### 3.2. Comparison of Injection Parameters

The statistical difference shows that the experimental group is less than the control group in the aspects of contrast volume, injection time, injection speed, saline chaser volumes, and flow rates. (*P* ＜ 0.05 for all). The specific data are shown in Table 2.

### 3.3. Objective Imagine Quality

There is no significant statistical difference between the experimental group and control group on right parasternal soft tissue. The difference in the aortic root, SD noise, SNR, CNR, and the proximal/mid/distal segments of three main branches of coronary vessels existed, and the experimental group is less than the control group in these aspects. The specific data are shown in Table 3.

### 3.4. Optimal Vascular Enhancement

The number of the three major vessels in the ideal vascular range (300–450HU) was counted, as shown in Table 4 and Figure 1*χ*2 value = 334.25, *P* = 0.001 < 0.05.

### 3.5. Comparison of Three Major Vessels with Aspects of BMI Subgroups

There exists a statistical difference between the experimental group and control group on the aortic root and segments of coronary vessels as expected (*P* < 0.05 for all). During the control group, the analysis turns out that the BMI≤20 subgroup differs from the 25 < BMI < 26 subgroup with the aspect of mid-RCA, (*P* = 0.026 < 0.05), on mid-LAD, and the BMI≤20 subgroup differs from 20 to 21，22∼23，and 25∼26 subgroups (*P* = 0.045,0.026,0.001). There was no statistical difference between BMI subgroups of the remaining vessels. The specific data are shown in Table 5, Figure 2. *∗* means statistical difference.

### 3.6. Subjective Imagine Quality

Using the Mann–Whitney *U* test， the subjective points between the two groups did not have a statistical difference. *Z* value = 0.394; *P* = 0.694 > 0.05. The specific data and intuitive presentation are shown in Table 6, Figure 3.

### 3.7. Impact of BW, BSA, and BV on Vascular Attenuation

In the control group with fixed 42 ml contrast volume, 3.5 ml/s injection speed, correlation analysis, and single linear regression showed that BW (body weight) has a medium negative correlation with vascular attenuation (*P* = 0.001＜0.05, *r* = −0.421) and aortic root attenuation (HU)  = −5*∗*BW (kg) + 948, *P* < 0.001. BSA (body surface area) has a medium negative correlation with vascular attenuation (*P* = 0.001, *r* = −0.457). Aortic root attenuation (HU) = −323*∗*BSA (m2)+ 1171 (*P* < 0.001); BV（blood volume） has a medium negative correlation with vascular attenuation (*P* ＜ 0.05, *r* = −0.477); aortic root attenuation (HU) = −86*∗*BV(L) + 1171, *P* < 0.001. The intuitive presentation is shown in Figure 4.

### 3.8. Analysis of Relationship between BMI, BW, BSA, and Blood Volume (BV)

Single linear regression shows that BV for male (L) = 0.077*∗*BMI (kg/m^2^) + 2.648, *P* < 0.001, *r* = 0.46; BV for female (L) = 0.083*∗*BMI (kg/m^2^) + 1.649, *P* < 0.001, *r* = 0.52.BV for male (L) = 0.042*∗*weight (kg) + 1.735, *P* < 0.001, *r* = 0.85; BV for female (L) = 0.046*∗*weight (kg) + 0.939, *P* < 0.001, *r* = 0.82; BV for male (L) = 2.788*∗* BSA (m^2^) −0.424, *P* < 0.001, *r* = 0.92; BV for female (L) = 2.971*∗*BSA (m2)−1.119, *P* < 0.001, *r* = 0.87. The intuitive presentation is shown in Figure 5.

A multiple linear regression model was used to predict vascular enhancement based on gender difference, BV, age, and heart rate.

A significant value was found (*F* = 14.942), with an *R*^2^ of 0.309. Vascular attenuation (Y) is equal to Beta0 - Beta1 (Sex) + Beta2 (Age) - Beta3 (Blood Volume) - Beta4 (Heart rate), among all the variables, BV was able to predict the attenuation individually (Table 7).

### 3.9. Explanation of the Feasibility of BMI Indicator by BV

The problem with using the BMI indicator is that it could not tell the difference in body size. The small body size could have the same BMI as the bigger one. However, the difference could be described by BV in which the correlation counts the most. In the control group， the study divided the male or female patients into high and low BV parts according to the median BV calculated. Male medium BV is 4.3 L, and female medium BV is 3.5 L. There exists a statistical difference between high and low BV groups (male *t* = 2.264, *P* = 0.028; female *t* = 4.419). Among the BV calculated, the population above the third quartile still meets the requirement: the description of aortic root attenuation was as follows: male (481 ± 80) HU and female (538 ± 108) HU(Figure 6).

## 4. Discussion

The present injection schedule makes the operator choose the fixed injective speed based on the selected tube voltage whatever the patients' weight (70KV−3.5 ml/s, 80KV−4 ml/s, 90KV−4.5 ml/s). The injective time equals scan time +7 s, which are often 11∼12 s. So injection volume could nearly seem as fixed under the single voltage. When the third-generation CT chooses low voltage (70/80 KV), the clinical question is whether the coronary enhancement of some patients is so high (>500HU) that degree of stenosis could be underestimated.

Although the CARE DOSE 4D of the third-generation DSCT including automatic tube potential selection and tube current modulation could make machine scanning factors vary according to patients' anatomy to determine the optimal combination [4], it is still uncertain about the influence of patients' individualized difference. The present study indicated that body weight, BMI, and other individual factors still have an effect on contrast enhancement, which corresponds to the conclusion made by Wang et al. [4]. Meanwhile, among all the indicators, the correlation of blood volume counts the most (*r* = −0.477). Unlike the strong correlation of body weight, body surface area, and so on without the CARE DOSE 4D [6], these indicators get a weaker correlation with the ‘disturbances' of changeable current.

Another important finding was that gender difference may have no obvious effect on attenuation based on the result of multiple linear regression. It is not strange that male patients have more blood volume than female ones with the same level of BMI/BSA/BW (Figure 5).

This is because female patients have more fat ratio than male ones and body fat is less vascular than visceral organs and muscles [8]. However, gender differences do not lead to the change of attenuation. One possible explanation was that female patients undertake higher tube currents than male ones. The finding of the current study does not support the previous research by Eijsvoogel [9], but his research was mixed with various levels of tube voltage which influence vascular enhancement. After all, there is no need to consider gender differences when ATVS selects 70 KV.

Mangold et al. [10]and Aschoff et al. [11] show that the CARE DOSE 4D tends to keep the signal-to-noise rate between different levels of tube voltage rather than signal. When tube current was beyond the machine's limitations, the technology tends to choose a higher level voltage and lower current to keep SNR stable. It is well known that a low tube voltage increases the attenuation of iodinated contrast agents [4] and the noise at the same time. Higher current and iterative reconstruction (IR) are used for decreasing the noise [11]. The requirement of contrast agents between different levels of tube voltage varies. So it is unsuitable to focus on individual factors to adjust the agent ignoring the effect of tube voltage and current. That is why the present study limits the 70 KV.

The BMI distribution range is 19∼26 during preexperiments when ATVS selects 70 KV. Among the injective parameters, iodine delivery rate (IDR) is a key element in vascular attenuation [8], so we designed the ladder-like low iodine delivery rate injection protocols to correspond to variations in BMI. One advantage is that the protocol could be operated easily. The volume value could be calculated as BMI value + 4, and the injection speed value could be calculated by volume/10s. On the contrary, using the BSA or BV as the indicator may result in large data redundancy. Such situation may not be suitable for busy clinical staff. We also adjust the saline chaser to 18 ml and 3 ml/s referring to the phantom study by Behrendt et al. [12].

The experimental group showed satisfying image quality as expected. Compared to the control group, the attenuation of the aortic root and three main branches of coronary vessels have decreased obviously. The number of ideal vessels counts more which reached the aim of the experiment. Meanwhile, the subjective image quality was not significantly different between these two groups. However, the noise of the experimental group is lower than the control group. The phenomenon could be attributed to population selection bias. Though there is no statistical difference in height, weight, or BMI between the two groups, the experimental group may get a higher average level of tube current which has a positive influence on attenuation (Figure 3 C1 C2). As the reduced injection agent is the main factor in decreasing attenuation, the two groups are still comparable. Another advantage of the new injection protocols is the reduction of the possibility of immediate hypersensitivity reactions (IHR) [13]. Compared to 42 ml of contrast agents in the control group, the average of 26 ml in the experimental group has been reduced by 38%. Though side reactions are infrequent, the lower injection volume and speed could be safer.

There is a large body of literature suggesting that BMI could be the indicator to adjust the injection protocols [4, 14]. Thus far, only a few studies have investigated the effect of BMI on vascular enhancement with the third-generation DSCT under a single voltage. However, the negative correlation between BMI and attenuation was not as strong as we expected. Such situation seemed to have conflicts with the high success rate in the experimental group. As the independent predictor, we tried BV to explain the phenomenon. People with different BV were divided into the same BMI subgroup resulting in the difference in attenuation. That is why the difference between our small BMI subgroups did not exist generally (Table 5). However, there still exists the trend that BMI and BV grow together (Figure 5(a)). As the sample size increases, we have reason to believe that the trend toward BMI and vascular enhancement will become clearer. We also conducted the patients in the experimental group above the third quartile BV whose images still meet the required CT value. After all, the step low flow rate and volume protocol are feasible.

The study also includes the BW and BSA toward attenuation. BW is the common clinical factor to adjust contrast agents with the ratio of 1 : 1. But similar to gender difference, the same weight with a different ratio of fat may result in different enhancement [15]. However, with the selection of the population by CARE DOSE 4D, it seemed suitable for BW to be an indicator. BSA is also a usual indicator to evaluate metabolic mass [6]. In our study, it corresponded to BV maximally. The point is the difficulty to operate in clinical practice which is similar to BV.

The present study has several limitations. First, We limit the tube voltage to 70 KV, meaning the miss of actual practice in other single voltage. Based on our experience, using the low flow and volume is feasible at 80 KV. But we still need enough samples. Second, we did not compare the diagnostic performance of CCTA versus invasive catheter angiography to detect the real degree of coronary artery stenosis. Third, the large size of patients needs further consideration to adjust the agents.

To conclude, it is feasible to use the ladder-like low flow and volume protocols when ATVS chooses 70 KV. The number of vessels within a suitable CT value range counts more. With the retention of image quality, the study reduced the contrast volume and injection speed which shall decrease the risk of IHR. Meanwhile, it is an easier and more practical way to operate compared to other indicators.

## Figures and Tables

**Figure 1:** Comparison of optimal vascular enhancement.

**Figure 2:** Comparison of aortic root attenuation between BMI subgroups.

**Figure 3:** A1∼3 showed three branches of coronary artery of a female patient (162 cm, 55 kg, BMI 21,0) with the injection of 42 ml, 3.5 ml/s; white arrow means calcified plaque; CT value of aortic root is 762HU which is believed too high. B1∼3 showed a female patient in the experimental group (166 cm, 57 kg, BMI 20.69)，with a volume of 24 ml, and a speed of 2.4 ml/s. The CT value of the aortic root is 524HU with a suitable range of enhancement on three main branches. C1 and C2 are two different male patients with 165 cm and 62 kg both, injected with 42 ml and 3.5 ml/s. C1's aortic root CT value is 711HU; tube current is 502/734 mAs; C2's CT value is 562HU; tube current is 366/734 mAs.734 mAs is a fixed tube current reference when tube voltage is selected at 70 KV.

**Figure 4:** Graphs show the distribution of aortic root enhancement plotted against body weight (a), body surface area (b), and blood volume (c). A medium negative correlation was observed between enhancement and BW(*r* = −0.421), BSA(*r* = −0.457), and BV(*r* = −0.477). Blood volume has the highest correlation. Ninety-five percent of CIs (dotted fitting lines) are fit to the regression line (solid fitting line). o = male patients, + = female patients.

**Figure 5:** Graphs show the distribution of blood volume plotted against BMI (a), BW (b), and BSA (c). A medium to strong positive correlation was observed between BV and BMI, BW, and BSA. Male patients have more blood volume than females. o = male patients, + = female patients.

**Figure 6:** Graphs A show that the low BV group has higher attenuation than the high BV group in the control group. Graph B shows that point A and point B have the same BMI in the control group, point A is a female patient with a height of 156 cm, weight of 55 kg, BV 3.35 L, and aortic root attenuation of 875 HU; point B is a male patient with the height 172 cm, weight 67 kg, BV4.6 L, and aortic root attenuation of 486 HU. Graph C shows that the patients above the third quartile BV in the experimental group still meet the requirement.

**Table 1:** Patients characteristics (‾*x* ± *s*).

		Experimental group	Control group	T/*Z*	*P*
Sex	Male	75	83	0.93^a^	0.335
	Female	65	57		
Age (years)		59.0 ± 11.6	61.3 ± 11.7	−1.841	0.068
Height (cm)		163.8 ± 7.2	163.7 ± 7.6	−0.110	0.902
Weight (kg)		60.5 ± 8.5	60.3 ± 8.3	−0.058	0.954
BMI (kg/m^2^)		22.50 ± 2.17	22.41 ± 2.37	−0.053	0.958
Heart rate (beats/min)		70.6 ± 9.3	71.1 ± 11.9	−0.632	0.527

**Table 2:** Comparison of injection parameters.

	Experimental group	Control group	*Z* value	*P*
Contrast volume (ml)	26 (4)	42	−10.20^a^	0.001
Injection speed (ml/s)	2.6 (0.4)	3.5	−10.29^a^	0.001
Injection time (s)	10	12	−11.83^a^	0.001
Saline chaser volume (ml)	18	40	−11.83^a^	0.001
Saline flow rates (ml/s)	3	4	−11.83^a^	0.001

a: calculated using the Wilcoxon rank sum test.

**Table 3:** Comparison as a whole.

	Experimental group	Control group	*T*/*Z*	*P*
Aortic root (HU)	523 ± 82	634 ± 87	−11.65	0.001
SD noise (HU)	28 ± 4	32 ± 5	−6.17^a^	0.001
Contrast tissue (HU)	123 ± 12	125 ± 15	−1.50	0.136
SNR	18.7 ± 3.5	20.3 ± 4.0	−3.22	0.001
CNR	14.3 ± 3.3	16.3 ± 3.7	−4.43	0.001
Proximal RCA (HU)	473 ± 90	642 ± 101	−16.53	0.001
Mid RCA (HU)	440 ± 98	612 ± 103	−15.09	0.001
Distal RCA (HU)	390 ± 94	581 ± 117	−15.33	0.001
Proximal LAD (HU)	491 ± 84	598 ± 93	−10.25	0.001
Mid LAD (HU)	440 ± 86	556 ± 93	−10.79	0.001
Distal LAD (HU)	363 ± 75	482 ± 94	−8.58^a^	0.001
Proximal LCX (HU)	478 ± 83	585 ± 96	−7.86^a^	0.001
Distal LCX (HU)	372 ± 80	485 ± 94	−11.07	0.001

a: Calculated using the Wilcoxon rank-sum test.

**Table 4:** Number of optimal vascular enhancement with comparison.

Vascular enhancement	Experimental group	Control group	Total
300–450HU	554	152	706
＜300HU/＞450HU	566	968	1534
Total	1120	1120	2240
*χ*2 value = 334.25, *P* = 0.001			

**Table 5:** Comparison with the unit of BMI subgroups.

Vessel segment	Group	≤20	20–21	21–22	22–23	23–24	24–25	25–26
Aortic root	Experimental group	537 ± 102	533 ± 89	494 ± 77	525 ± 65	530 ± 81	540 ± 68	504 ± 90
	Control group	690 ± 84	618 ± 104	624 ± 89	636 ± 55	624 ± 65	650 ± 89	598 ± 98
	t	−5.65	−3.25	−4.45	−6.48	−4.47	−3.88	−3.65
	P	0.001	0.004	0.001	0.001	0.001	0.001	0.002

Proximal RCA	Experimental group	485 ± 101	490 ± 84	444 ± 85	471 ± 78	480 ± 90	496 ± 87	448 ± 99
	Control group	705 ± 115	628 ± 123	630 ± 82	632 ± 62	651 ± 77	647 ± 84	599 ± 127
	t	−6.95	−5.03	−6.59	−8.04	−6.89	−5.09	−6.05
	P	0.001	0.001	0.001	0.001	0.001	0.001	0.001

Mid-RCA	Experimental group	444 ± 114	438 ± 83	433 ± 94	441 ± 82	441 ± 93	475 ± 107	410 ± 113
	Control group	681 ± 107	603 ± 136	582 ± 106	614 ± 80	629 ± 59	615 ± 83	564 ± 106
	t/*Z*	−6.60	−5.45	−4.80	−6.75	−9.33	−3.80	−3.77^a^
	P	0.001	0.001	0.001	0.001	0.001	0.001	0.001

Distal RCA	Experimental group	395 ± 74	357 ± 75	392 ± 109	398 ± 86	389 ± 80	423 ± 126	380 ± 100
	Control group	619 ± 124	565 ± 147	553 ± 130	596 ± 93	575 ± 92	619 ± 94	545 ± 123
	t	−7.21	−8.09	−3.80	−6.76	−6.92	−4.61	−5.27
	P	0.001	0.001	0.001	0.001	0.001	0.001	0.001

Proximal LAD	Experimental group	506 ± 90	480 ± 90	471 ± 90	491 ± 71	515 ± 84	518 ± 62	458 ± 87
	Control group	638 ± 104	585 ± 109	603 ± 86	590 ± 69	593 ± 69	647 ± 95	558 ± 104
	t	−4.46	−3.12	−4.10	−5.20	−3.42	−3.48	−3.88
	P	0.001	0.006	0.001	0.001	0.003	0.002	0.001

Mid-LAD	Experimental group	444 ± 114	438 ± 83	433 ± 94	441 ± 82	441 ± 93	475 ± 107	410 ± 113
	Control group	610 ± 97	552 ± 96	559 ± 77	546 ± 76	557 ± 89	560 ± 102	507 ± 97
	t	−5.04	−4.66	−4.76	−4.45	−4.31	−2.32	−3.75
	P	0.001	0.001	0.001	0.001	0.001	0.032	0.001

Distal LAD	Experimental group	359 ± 80	345 ± 63	342 ± 91	366 ± 77	362 ± 64	392 ± 73	377 ± 75
	Control group	529 ± 97	471 ± 104	455 ± 92	494 ± 63	475 ± 84	484 ± 126	467 ± 74
	t/*Z*	−5.60	−4.75	−3.30^a^	−5.41	−4.71	−2.68	−4.21
	P	0.001	0.001	0.001	0.001	0.001	0.015	0.001

Proximal LCX	Experimental group	483 ± 84	472 ± 76	446 ± 90	482 ± 70	498 ± 91	506 ± 72	464 ± 94
	Control group	633 ± 135	565 ± 95	567 ± 88	588 ± 69	582 ± 72	592 ± 95	565 ± 95
	t/*Z*	−4.20	−4.04	−3.89	−5.38	−2.65^a^	−2.82	−4.00
	P	0.001	0.001	0.001	0.001	0.008	0.011	0.001

Distal LCX	Experimental group	393 ± 94	354 ± 64	334 ± 97	382 ± 76	373 ± 64	393 ± 71	374 ± 78
	Control group	497 ± 127	477 ± 103	487 ± 90	479 ± 96	493 ± 78	486 ± 76	472 ± 91
	t	−2.90	−5.11	−5.14	−3.61	−5.21	−3.39	−4.97
	P	0.009	0.001	0.001	0.002	0.001	0.003	0.001

a: using the Wilcoxon rank-sum test. A difference exists in mid-RCA and mid-LAD of the control group. Mid-RCA Dunnett's T3 test shows that BMI ≤ 20 subgroup differs from the 25 to 26 subgroup (*P* = 0.026 ＜ 0.05). LSD method shows BMI ≤ 20 subgroup differs from 20 to 21, 22–23, and 25–26 subgroups of mid-LAD (*P* = 0.045, 0.026, 0.001).

**Table 6:** Subjective image quality comparison.

Point	Diagnostic segments of coronary artery			4 point
	1 point	2 point	3 point	
Experimental group	1005	102	2	3
Control group	1011	90	7	4
*Z*	0.394			
*P*	0.694			

Note: data are numbers of segments, and data in parentheses are percentages.

**Table 7:** Multiple linear regression analysis: the effect of variables.

Variables	Beta	Beta^*∗*^	Estimate	|*T*|	*P*	95% CI for estimated
Constant	*β*0		982.679	7.72	0.001	[730.7 to 1234.7]
Sex	*β*1	−0.086	−17.706	0.78	0.440	[−62.5 to 27.1]
Age (years)	*β*2	0.276	2.338	3.65	0.001	[1.1 to 3.6]
Blood volume (L)	*β*3	−0.502	−91.298	4.58	0.001	[−130.8 to −51.8]
Heart rate (times/min)	*β*4	−0.164	−1.393	2.18	0.032	[−2.7 to −0.1]

*∗*: Standard beta *R*^2^ = 0.309.

## Data Availability

The data and materials during the current study are available from the corresponding author on reasonable request.
